# Innovative Design of a Healthy and Environmentally Friendly Intelligent Cleaning Robot in a Smart City Public Environment

**DOI:** 10.1155/2022/1602125

**Published:** 2022-08-21

**Authors:** Chang Wei, Peng Wang, Yiming Ma, Ruoxi Li

**Affiliations:** ^1^School of Arts and Media, Suqian University, Suqian, China; ^2^Coventry University, Coventry, UK; ^3^Nanjing Institute of Technology, Nanjing, China; ^4^Fujian University of Technology, Fuzhou, China

## Abstract

With the expansion of modern society, there has been a substantial increase in the number of structures with multiple stories. Skyscrapers are not only the dream of incredible architects that desire to command the sky, but they have also transformed and defined how we live in the modern day. Building walls, on the other hand, are constantly affected by acid rain, dust and mist, meteorites, and bird droppings since they are exposed for lengthy periods of time. Furthermore, the challenges of cleaning at great heights are becoming increasingly critical. Figuring out how to most efficiently maintain the outside surfaces of skyscrapers so as to extend their longevity, as well as their worth in urban contexts, is a major concern for the health and cleanliness of the public environment in modern cities. The creation of “smart cities” offers a huge opportunity to achieve this goal. A PLC control system for an intelligent cleaning robot was presented in this study, together with its wire design, control demands, hardware selection, and control system. Furthermore, it provided a design for a cleaning robot that would operate within the context of a smart city. A PLC system would be used in this design to detect the cleaning position and initiate automatic cleaning. The operation of the system revealed that the PLC-based intelligent cleaning robot control system has high dependability, strong operating efficiency features, and a high promotional value.

## 1. Introduction

In November of 2008, IBM was the first company to unveil its “Smart Planet” initiative. The swift advancement of society, economy, and information technology has inexorably led to the rise of “smart cities” all over the world at the same time that these places are undergoing the process of urbanization [1]. The potential and methodology of smart cities are two of the most interesting aspects of these urban developments. In order to accomplish intelligent administration of cities through scientific analysis of data on urban development and to make urbanization more comprehensive and environmentally friendly, [2] they are working toward this goal.

The external glass of high-rise buildings is subjected to the elements, including the sun and rain, for extended periods of time. This exposure results in the accumulation of dirt and wear and tear, which has a detrimental effect not only on the structural integrity of the building but also on the aesthetic appeal of the surrounding area. This has a negative impact on the life expectancy of the building in addition to having an aesthetic impact on the city. Due to this, it is absolutely necessary to clean the glass of high-rise buildings when the facade cleaning industry is once again on fire; yet, operating at great height involves problems for both the equipment and the personal safety of the workers.

As smart cities and networks are built, technology is revolutionizing how buildings are cleaned, and the overall environment for public health is becoming more intelligent. This transformation is taking place concurrently. Drones and robots are undergoing this transformation as well. To make a big impact in Spiderman's work, it is vital to design robots with technological breakthroughs [3].

As a result of the current state of aerial cleaning in China, on the one hand, there are no applicable laws and regulations to guide this industry, and on the other hand, businesses are unwilling to invest in excessive equipment and money, which results in aerial cleaners having rudimentary equipment and leading to a high number of accidents. In modern times, the most frequent types of cleaning techniques for facades are physical and chemical [4]. The use of water in physical procedures is typically limited to rinsing or spraying, but these processes waste an enormous amount of water and are not good for the environment. In addition, high-pressure water pistols can easily break the glass, and they are unable to remove some stains that are particularly tenacious. In its most basic form, chemical cleaning refers to the process of removing dirt from the surface of a building by making use of various chemical reagents. The primary component of the cleaning agent is a neutral liquid; nevertheless, the pH value of the liquid is not neutral; rather, it is either slightly alkaline or slightly acidic. Glass that has been used for an extended period of time may become damaged, which may lead to pollution of the surrounding environment. Consequently, it is necessary to develop an intelligent robot that can clean glass while it is suspended.

This design took the concept of smart cities and combined it with the requirements of building facade cleaning. The goal was to investigate and rationally screen the characteristics of healthy and environmentally friendly cleaning robot equipment and functions so that they could be tailored to meet the needs of cities and tall buildings. In addition, the design incorporated a broad spectrum of expertise and technology, in addition to the logical selection and application of materials, in order to address quality and structure at all levels, avoid the possibility of technical drawbacks, carry out reasonable calculations, and effectively address issues such as precise spot cleaning.

It connected items based on smart cities; cleaned skyscraper facades efficiently and conveniently to maximize economy, health, and environmental protection; and solved a large number of issues that skyscrapers encountered in smart cities.

## 2. Trends and Developments in Intelligent Cleaning Robots

In a smart city, the most recent information technology is used to its full potential in order to connect a variety of different things with the assistance of the Internet of Things. A smart city also relies on cloud computing and intelligent mobile terminals' extensive data analysis platforms for the purpose of data analysis [5]. It does this by monitoring, analyzing, integrating, and intelligently responding to situations; combining efforts to open up smooth interconnection pathways; integrating and optimizing existing municipal resources; and bolstering construction, management, and service delivery in urban planning. All of these functions are integrated using this method. Accelerated urbanization is frequently accompanied by a number of other so-called “urban diseases,” which can include population explosion, housing issues, environmental harm, and transportation congestion. The development of smart cities has become a standard requirement and a significant trend in the development of countries around the world in order to solve problems of this nature and to promote urban development that is healthy, safe, and sustainable. This is why the development of smart cities has become so important. The concept of smart cities is gaining popularity all over the world, and China is one of the countries that is leading the pack in this area. The unmanned aerial vehicle (UAV) sector is now experiencing explosive growth and has found applications in a variety of fields, including the military and agriculture. The range of missions that can be carried out by uncrewed aerial vehicles has significantly broadened as a result of the development of UAVs with airborne operational capabilities [6].

Cities are becoming more aware of the significance of facade cleaning because the appearance of a building's façade can provide insight into the general public's perception of both the business and the city. Even legislation mandating regular facade maintenance has been enacted in a number of places across the country. The fact that the skyscraper is situated in the middle of the city, however, leaves it exceptionally polluted in relative terms. Because of the stone's absorbency, pollutants from the air, dust, acid gas in the air, and the exhaust from steam locomotives accumulate on its surface. Acid rain hastens the dissolution of these pollutants from the stone and causes them to become absorbed in the capillary pores of the stone, which makes it more difficult to remove stains from the stone. These pollutants build up more quickly and are more difficult to remove, particularly in the case of flamed stone; also, professional cleaning products will be unable to get rid of them [7].

### 2.1. The Significance of Healthy and Environmentally Friendly Intelligent Cleaning Robots in Public Environments in Smart Cities

On the one hand, the cleanliness of a high-rise structure is a representation of the appearance of the city, and on the other hand, it indicates whether or not the public health of the city is up to standard. The rate of urbanization is increasing, which means that the outside surfaces of high-rise buildings in cities are exposed to more pollution throughout the year, making them subject to pollution from the air, dirt, and rainwater. These exposed surfaces have the potential to collect stains and lose their luster, which can have a negative impact on the building's overall look and perhaps cause erosion damage. Traditional manual cleaning methods, sometimes known as “spiderman” work, are currently the methods of choice for maintaining the facades of tall buildings, despite the fact that this task is becoming increasingly difficult to perform. The work is hazardous, and there is no assurance that safety will be maintained. In spite of the fact that the cleaning tools and equipment are very straightforward, the cleaners are required to carry buckets of water while also utilizing brush strips and rubber scrapers in order to complete the cleaning operation at great heights, washing areas downward as they go.

Manual cleaning is straightforward and adaptable, but it is ineffective, expensive, and fraught with significant danger. In a more technologically sophisticated future, this will, without a doubt, be replaced by brand new cleaning robots. Cleaning robots play an essential part in both day-to-day living and the applications used in industry. These robots save both time and money on labor costs, in addition to freeing humans from tedious and repetitive cleaning tasks. It is a widely held belief that the development and establishment of smart cities have created the social conditions for the development of intelligent cleaning robots that are both healthy and environmentally friendly, and that make use of modern information technology to effectively manage and clean exterior walls. There is already some room for the design of cleaning robots that are suitable for the secure usage of outside wall cleaning [8]. This is due to the continual development of relevant technologies in the field of intelligent interaction in China.

This design, which was based on earlier research, suggested the concept of an intelligent cleaning robot that would be healthy, sustainable, and friendly to the environment as part of the smart city. A programmable logic controller (PLC) was what made it possible for the robot to recognize the cleaning position and perform automatic cleaning. PLC-based intelligent cleaning robot control system was found to exhibit high reliability, strong working efficiency, and other characteristics as a result of actual usage of the system. Additionally, it was found that the system, in all aspects, had specific innovative and research value that would enable it to meet the demands of the cleaning industry further and enhance its practicality.

### 2.2. Current Status of Research on Intelligent Cleaning Robots

Since the early 1980s, numerous researchers from both the United States and other countries have conducted research on cleaning robots, and as a result, several results have been acquired. The issue, on the other hand, is that of the many different kinds of cleaning robots that are currently available, only a limited number of robots are designed specifically to clean the façade of high-rise buildings. Despite this, only a very small fraction of the several varieties of cleaning robots are intended to clean the exterior surfaces of high-rise structures.

Depending on the setting in which they are deployed, several types of cleaning robots can be categorized as either being designed for usage in the home or a commercial setting. The most common types of cleaning robots can be broken down into the categories depicted in Figure 1. The particular setting in which these devices are deployed can also have an effect on the ways in which they perform their jobs and the modes in which they operate. The primary role of residential robots is to sweep dust and grime off of the floors; however, the big cleaning robots used in large public areas can also spray water, collect sewage, gather minor trash, and perform a variety of other duties. Manual and automatic modes of operation are also available to the user [9].

The creation of high building facade cleaning robots is now being worked on by prominent educational institutions, research organizations, and technological corporations from both the United States and other countries. The majority of these robots are still in the process of being developed and tested in laboratories. They have immature technology and a slow market penetration process, both of which are hampered by the difficult floor environment and the lengthy operation.

Conventional roller brush brushing and touch crawling actions are the defining characteristics of traditional facade cleaning robots. Sensitive sensors, a more complicated mechanical design, and a sound control system are required in order to do contact crawling. This can be accomplished with wheeled, footed, or tracked suction cups. There is some usefulness in contact motion for technological research, but its application in the real world is restricted. The cleaning effect of the roller brush is negatively impacted both by its slow speed and its limited number of brushing cycles. Because of both its size and structure, it is relatively massive and bulky, which can have a negative impact on its smoothness [9, 10].

The majority of the wall climbing robots that have been deployed for stair cleaning in China in recent years have been utilized in conjunction with predetermined tracks for the purpose of cleaning. Leatu Robotics has developed a facade cleaning robot that is able to automatically clean glass walls up and down by lifting and line planning. This robot was created by Leatu Robotics. However, wall cleaning devices that use drones have not yet been invented, and their flexibility and unlimited access have not yet been utilized; as a result, there is now a gap in the market for drones around the world [11, 12] (see Figure 2).

### 2.3. Analysis of the Working Environment and Functional Requirements of Intelligent Cleaning Robots

The vast majority of cleaning robots are designed to operate in a wide variety of settings, both indoors and outdoors. These settings include numerous locations that are difficult or impossible to reach by hand. This design is only concerned with discussing the cleaning of building walls in outside conditions.

Large expanses of glass, stone, and sometimes even other materials make up the usual composition of the facades of modern buildings. When it comes to cleaning the facades shown in Figure 3, there are a number of aspects that are inconvenient. Due to the limitations of cleaning instruments, traditional hand cleaning is inefficient, time-consuming, and expensive. This is because traditional cleaning targets facades and glass. In addition, the task of the cleaning team is risky, and puts them at risk for injury when they are cleaning at great height.

Analyzing the cleaning environment is the first thing that needs to be done in order to create a healthy and environmentally friendly cleaning robot. This will ensure that the robot will be able to deal with the environment and fulfill its functional requirements [13]. The majority of the city's residential, office, and commercial buildings range in height from 60 meters to 100 meters, while structures that are taller than 150 meters are very uncommon. The city is home to a large number of residential, office, and commercial structures. In the beginning, it was decided that the working environment would focus on buildings that were less than 150 meters tall. The design presented the following functional needs, taking into consideration the surroundings of the roof, floor, and ground level of the tall building:

1. The floor is uneven; thus, the cleaning robot needs to be able to move up and down as well as side to side.
2. The robot has a high level of cleaning capability and improved environmental adaptation, making it suitable for a wide variety of exterior wall surfaces.
3. The robots are capable of crossing ordinary floor crossbar obstacles in a reliable manner.
4. The robot's responsiveness, stability, and reliability are ensured by effective communication and control management between the robot and the ground.

## 3. Health and Environmental Protection Type Intelligent Cleaning Robot Design Analysis

According to the actual working environment and functional requirements, the overall design plan was initially determined, a specific design workflow analysis was carried out, and the overall system design was planned according to the designed workflow, which was divided into hardware system design and exterior modeling design.

### 3.1. Analysis of the Working Process of an Intelligent Cleaning Robot

In order to design an intelligent cleaning robot, it was essential first to understand how it works simply. The working process of a cleaning robot could be broken down into several steps. The working area was first sprayed with water to facilitate the dilution of the cleaning agent; then the cleaning agent was sprayed; the roller brush was repeatedly rolled and rubbed to remove dirt and grime; and finally, the surface was rinsed clean again with water. The working steps are shown in Figure 4 [14].

(1) Task analysis.

The cleaning robot started working when the user gave the start command. Initially, the sensors detected the range to be cleaned, and once that range was detected as being in the scrubbing range, the bottom contactors opened, the detergent and water valves worked, and the cleaning began. When the floor gave the end command, the cleaning robot closed all contactors and valves and ended the cleaning [15].

(2) Flow chart.

Based on the above analysis, Figure 5 illustrates the workflow of the intelligent cleaning robot.

## 4. Healthy and Environmentally Friendly Intelligent Cleaning Robot Design Concept

Several factors, including the high cost of manual operation and the low level of safety associated with working at heights, impede the development of high-level cleaning. In order to improve the public health environment of cities, we must focus on solving these problems to improve the cleaning rate of high-rise buildings [16, 17]. On this basis, a healthy and environmentally friendly intelligent cleaning robot was proposed to solve many of the problems of high-rise cleaning, in conjunction with the general trend of smart city development. The design concept was based on cleaning the façade of tall buildings with an intelligent and humane focus, supported by technologies such as precise positioning and robotics, on providing a safe, convenient, and reliable aid for tall building cleaning.

### 4.1. Design Concept of the Intelligent Cleaning Robot System

The system control requirements are shown in Figure 6.

### 4.2. Control Hardware Design

As an internationally recognized German company, Siemens produces highly commendable programmable controllers in various applications, including chemical processing, machinery, and first-line production lines.

The Siemens S7 series PLCs are easy to use, can be processed quickly, have strong network communication capabilities, and are highly reliable when used in cleaning robots, as shown in Figure 7.

The PLC controller of the S7-200 series and the expansion module of the EM235 was chosen for this design, as shown in Figure 8.

### 4.3. Motor and Drive Control

DC motors are rotating motors that convert direct current into mechanical energy, and are widely used in small appliances or electronic equipment such as electric shavers, hairdryers, electric toys, and electronic watches. They are characterized by good speed regulation, easy starting, and the ability to start with a heavy load, which is why they are still widely used.

The asynchronous motor, also known as an induction motor, is a type of AC motor. With a simple structure, uncomplicated manufacturing process, low price, and long life, asynchronous motors are widely used in water pumps, machine tool grinders, compressors, fans, household appliances, medical equipment, and other fields.

Synchronous motors are also AC motors mainly used in large machines, such as water pumps and blowers.

As a result of considering various factors, including application and price, efficiency, lifetime, and practical laboratory considerations of the three types of motor—DC motor, asynchronous motor, and synchronous motor—asynchronous motors were more suitable for the design of cleaning robot systems (see Figure 9).

### 4.4. Selection of Detection Elements

Even though modern sensors may appear similar, they differ in principle and structure, and we must choose the appropriate sensor according to the environment in which the robot will be operating. The choice of the sensor would have a significant impact on the accuracy of the measurement.

### 4.5. Battery Selection

Lithium iron phosphate batteries are a fantastic choice when it comes to the usage of batteries for cleaning robots because of their low weight, resistance to humidity, high capacity, and long life. In addition to the one-of-a-kind conditions under which the robot was designed to do its tasks, it was essential that a solar panel be mounted on the body of the device in order to ensure its durability and serve as a secondary source of power.

## 5. Innovative Design Practice of a Healthy and Environmentally Friendly Intelligent Cleaning Robot

Based on the work in the previous chapters, a workflow was set up, and motors and electronic components were selected. The design was intended to explore a new path for a high-rise façade cleaning robot through the combination and improvement of a cleaning robot and a flying drone, which could break the limitations of the lack of crucial functions, such as the ability to clean various façade materials independently [12, 18].

In order to meet the needs of intelligent city construction, a healthy and environmentally friendly cleaning device has been designed to clean all types of different façade materials through simulation and data detection. The product and the interactive process were implemented scientifically, operationally, efficiently, and unobstructed [19, 20].

### 5.1. Sketching

After selecting the operating principle and the motor, the design was brainstormed and is shown in Figures 10 and 11. Figures 10 and 11 illustrate the product's various parts, details, and overall structure.

### 5.2. Digital Modeling Design

The appearance of the virtual model was designed using digital modeling techniques based on existing sketches, as shown in Figure 12.

### 5.3. Foam Modelling

A 1 : 1 foam model was created using foaming material to test the suitability of the 3D printed model in a real-life scenario, skipping the paper mold because of the product's specificity and the structure's complexity. This test was carried out by measuring the dimensions and thickness of the foam model to determine the dimensions of the final model (see Figure 13).

### 5.4. Physical Model Presentation

Figure 14 illustrates the results of testing the 3D printed model on a site such as a glass curtain wall.

Figure 15 shows the cleaning robot at work in the hot sun in a photograph of an actual building in Nanjing and a product rendering.

## 6. Conclusion

As a result of this research, design solutions have been proposed and determined by combining an evaluation of the present market position for cleaning robots with high-rise facade cleaning requirements. The study concentrated on high-rise buildings in particular. From the overall design to the detailed design, modeling, debugging, and optimization, we gained a better understanding of the social significance of high-rise cleaning, as well as a better understanding of today's cleaning robots, as well as some regrets and problems that could be identified from the previous research results. Furthermore, we obtained a deeper knowledge of the societal relevance of high-rise cleaning as well as of today's cleaning robots.

The market for aerial cleaning is gaining traction among both domestic and foreign businesses, and intelligent robots created exclusively for aerial cleaning are becoming more readily available. However, we can observe that aerial cleaning robots are not frequently deployed. One of the key reasons for this is the price of existing items, which ranges between $100,000 and $200,000 USD. The equipment is overly bulky, and its use needs the installation of an awkward track. A large number of technological companies and teams are attempting to develop viable high-altitude cleaning robots. However, many technologies are still in the early stages of development, and many domestic businesses are claiming ideas made by multinational organizations. Given that high-altitude intelligent cleaning robots are yet to be mass-produced or employed on a large scale, more research into their design and development is required. As a result, in order to fill the gap in China's intelligent cleaning market, the country must develop its own brand of cleaning robots. Home cleaning robots and those utilized in Europe, the United States, and other countries have a large technological gap. This is primarily due to the fact that domestic cleaning robots have a relatively simple design, are not widely used, and have ineffective support technologies. In this article, Siemens S7-200 series PLCs were used to design the cleaning and cleaning device system so that the cleaning route could be more reasonable, and the machine could complete its task efficiently and in the shortest amount of time. This was done so that the machine could do its duty efficiently and quickly.

## Figures and Tables

**Figure 1:** Table of cleaning robot types.

**Figure 2:** Development of a façade cleaning robot by Leatu Robotics.

**Figure 3:** Common materials used in building facades.

**Figure 4:** Step-by-step diagram of the cleaning robot's work.

**Figure 5:** Workflow diagram.

**Figure 6:** System schematic.

**Figure 7:** Basic configuration and performance diagrams of S7-22 ^*∗*^ series CPUs.

**Figure 8:** EM235 parameters.

**Figure 9:** Motor parameters.

**Figure 10:** Brainstorming dispersion keywords.

**Figure 11:** Sketch.

**Figure 12:** Virtual modeling.

**Figure 13:** The process of making a foam model.

**Figure 14:** Physical model.

**Figure 15:** Actual view.

## Data Availability

The dataset used to support the findings of this study are available from the corresponding author upon request.
